# Low Power Scheduling Approach for Heterogeneous System Based on Heuristic and Greedy Method

**DOI:** 10.1155/2022/9598933

**Published:** 2022-06-26

**Authors:** Junke Li, Bing Guo, Kai Liu, Jincheng Zhou

**Affiliations:** ^1^School of Information Engineering, Suqian University, Suqian, Jiangsu 223800, China; ^2^School of Computer and Information, Qiannan Normal University for Nationalities, Duyun, Guizhou 558000, China; ^3^Jiangsu Province Engineering Research Center of Smart Poultry Farming and Intelligent Equipment, Suqian, Jiangsu 223800, China; ^4^College of Computer Science, Sichuan University, Chengdu, Sichuan 610065, China; ^5^Key Laboratory of Machine Learning and Unstructured Data Processing of Qiannan, Duyun 558000, China; ^6^Key Laboratory of Complex Systems and Intelligent Optimization of Guizhou, Duyun 558000, China

## Abstract

Big data, cloud computing, and artificial intelligence technologies supported by heterogeneous systems are constantly changing our life and cognition of the world. At the same time, its energy consumption affects the operation cost and system reliability, and this attracts the attention of architecture designers and researchers. In order to solve the problem of energy in heterogeneous system environment, inspired by the results of 0-1 programming, a scheduling method of heuristic and greedy energy saving (HGES) approach is proposed to allocate tasks reasonably to achieve the purpose of energy saving. Firstly, all tasks are assigned to each GPU in the system, and then the tasks are divided into high-value tasks and low-value tasks by the calculated average time value and variance value of all tasks. By using the greedy method, the high-value tasks are assigned first, and then the low-value tasks are allocated. In order to verify the effectiveness and rationality of HGES, different tasks with different inputs and different comparison methods are designed and tested. The experimental results on different platforms show that the HGES has better energy saving than that of existing method and can get result faster than that of the 0-1 programming.

## 1. Introduction

As an important driving force of social development and world economic growth in the 21st century, ICT (information and communication technology) industry consumes 10% of the global power consumption [1], and its total carbon emissions account for 2%–2.5% of the total global carbon emissions, especially in developed countries, reaching 10% [2]. The Intergovernmental Panel on Climate Change of the United Nations has released a report, pointing out that if the temperature of global warming is to be limited to 1.5°C higher than that before the Industrial Revolution, unprecedented changes are needed, efforts should be made to completely stop using fossil fuels by 2050, and zero carbon emissions should be achieved [3]. In order to promote the sustainable development of ICT industry, green computing [4–12] has become the consensus of many researchers at home and abroad. At present, ICT industry represented by big data technology and artificial intelligence technology is constantly changing our life, transportation, learning, and cognition of the world, which makes the heterogeneous computing system (HCS) based on GPU (graphics processing unit) supporting the development of these technologies become the mainstream of computer system. The characteristics of GPU heterogeneous system such as high acceleration, easy to learn, and easy to expand make it develop rapidly. At present, it is widely used in big data processing, deep learning, cloud computing, artificial intelligence, unmanned vehicle driving, molecular simulation computing, and other fields. The huge application market also has greatly promoted the development of GPU heterogeneous system. In a typical GPU heterogeneous system, CPU usually allocates computing tasks to GPUs for calculation; in a computer system composed of multiple GPUs, how to allocate computing tasks to each GPU will greatly affect the power consumption of the whole system [13–35]. In this paper, the low power task scheduling of GPU heterogeneous system is studied. Although the performance and power of GPU heterogeneous system are greatly improved than that of traditional computer system, its power consumption is still high in the whole computer system. In order to comply with the development of ICT industry, the power optimization of GPU heterogeneous system should be studied in depth.

For reducing the power consumption of HCS, scholars have put forward various methods and models, but there are some problems in the current research work; for example, it is necessary to manually rewrite the target task code [13, 19], the energy consumption of heterogeneous systems is affected by the order of task execution [32, 34], and assuming that the power of GPU is constant when the tasks run [30], and it is necessary to run the task in advance to obtain the parameters [12, 26] before the task is scheduled. In order to effectively alleviate the above problems and make HCS more widely adapt to the diversity of tasks, this paper mainly focuses on the energy saving of heterogeneous systems with multiple identical GPUs. Inspired by the 0-1 programming, the HGES (heuristic and greedy energy saving) scheduling model is proposed by using heuristic and greedy method. The model first obtains the power consumption and time of the tasks on each GPU, and then the energy optimization problem is transformed into a scheduling problem. HGES consists of the following steps:

1. Power measurement and task execution time acquisition: HIOKI3334 power meter is used to obtain the energy consumption of the task by measuring the current and voltage. This study does not change the running time of the task, so the running time of the task is the actual running time of the task in the experimental environment.
2. Task scheduling: in the environment of multiple identical GPUs, the average power consumed by randomly processing a certain number of tasks is the same. The difference lies in the speed of the overall execution time. Therefore, the problem of energy saving can be transformed into the problem of time minimization. In this paper, HGES method is designed to solve the problem.
3. Verification: in order to verify the effectiveness of HGES. First, analyze its performance. Then, its effectiveness, rationality, and feasibility are verified by experiments.

The contributions of this paper are as follows:

1. This paper analyzes the essence of energy saving problem in heterogeneous systems with multiple identical GPUs and transforms it into scheduling problem.
2. Based on the 0-1 programming, HGES scheduling method is proposed by heuristic and greedy method. It calculates the average time and variance of all tasks to be executed according to the time of task execution and then divides all tasks in each GPU into high-value tasks and low-value tasks according to average value and variance; after sorting the high-value tasks, greedy method is used to assign the high-value tasks first and then the low-value tasks.
3. The experimental results show that the HGES method on different platforms can save more energy than that of existing methods. Compared with 0-1 programming method under best solution, HGES can get result faster.

The rest of the paper is structured as follows.  Section 2 shows related works; heuristics from 0-1 programming are introduced in Section 3; Section 4 presents the HGES method; our proposed method is verified and compared in Section 5; Section 6 summarizes the work of this paper.

## 2. Related Works

The research on energy saving in task scheduling can be divided into two categories: energy saving scheduling technologies based on task characteristics and energy saving technologies for task scheduling. They are described in detail as follows.

The first is energy saving scheduling technology based on task characteristics. [9, 10] point out that the storage requirements of tasks, task migration, and the improvement of scheduling strategy are helpful to the improvement of system performance. Based on this, Zhan et al. [11] research the energy optimization of hybrid scratchpad memory which consists of SRAM and nonvolatile memory. Then, they propose data allocation for energy optimization which is composed of program analysis stage and data allocation stage. After the GPU supports the concurrent kernel execution feature, it provides a solution for energy saving technology. Li et al. [12] have obtained the parameter *R*_*i*_ by running the CUDA profiler tool in advance to determine the kernel category and have used the complementary characteristics of the task category as inspiration to implement concurrent kernel execution for energy saving. Jiao et al. [13] have proposed a static estimation power-performance model by using the method of predicting the ratio of block number, and it has guided energy saving of GPU by establishing the relationship between the ratio of block number and energy consumption among concurrent kernels; however, this method requires to convert task code. Inspired by the implementation of energy saving with complementary characteristics of task categories by [12], Li et al. [14] use the established energy saving regression prediction model and scheduling method to achieve the goal of energy saving after classifying tasks. Li et al. [15] have compared the energy consumption of the concurrent kernel and the sequential kernel, and choose a way to perform tasks with less energy consumption; for the acquisition of energy, the energy estimation model and the performance estimation model are used. Wen et al. [16] have proposed a graph-based algorithm to schedule co-run kernel in pairs to optimize the system performance. Workloads are represented by a graph (vertices stand for distinct kernels, while edges between two vertices represent the corresponding two kernels and co-execution can deliver a better performance than run them one after another). Edges are weighted to provide information of performance gain from co-execution. Wen and Oboyle [17] have proposed a runtime framework to detect whether to merge OpenCL kernels or to schedule them to the most appropriate devices separately by using a prediction model based on machine learning at runtime, so as to schedule multi-user OpenCL tasks to the most appropriate devices in heterogeneous systems.

The second is the energy saving technologies for task scheduling. Compared to a uniprocessor, multiprocessors have been shown to reduce the power problem. For saving energy of multi-processor architectures, task migration is an effective method. Based on this, Rupanetti and Salamy [18] propose a three-part framework to reduce energy which is task allocation technique, task migration, and task scheduling scheme based on the earliest deadline first method. Liu and Luk [19] obtain the task and processor resource parameters by running tasks in advance and then use the linear programming to achieve energy saving scheduling of LINPACK program in each processor, but this method requires manually rewriting the code of the target processor. According to the analysis method proposed by [21], Barik et al. [20] obtain the task characteristics and execution time parameters to adjust the load rate for achieving the purpose of reducing energy consumption of processor. After that, Ma et al. [22] have proposed a two-layer energy management framework with dynamic allocation layer and frequency regulation layer, compared four dynamic allocation schemes, and analyzed their advantages and disadvantages. Li et al. [23] point out the deficiency of researches on the energy and thermal issues of real-time applications with precedence-constrained tasks on heterogeneous systems and then propose both energy/thermal-aware task scheduling approach by assigning tasks in an energy/thermal-aware heuristic way and reducing the waiting time between parallel tasks. Bansal et al. [24] combine both the dynamic voltage scaling (DVS) and dynamic power management (DPM) techniques to save energy while scheduling preference-oriented fixed-priority periodic real-time tasks and then propose preference-oriented energy-aware rate-monotonic scheduling and preference-oriented extended energy-aware rate-monotonic scheduling algorithms to maximize energy savings while fulfilling preference value of tasks. Silberstein and Maruyama [25] have considered the energy of tasks on each processor, and they construct a minimum energy consumption scheduling method for multiple interdependent tasks according to the directed acyclic graph and verify the feasibility of the method when the processor has no overhead. Jang et al. [26] have studied the energy optimization of single task in multi-processor environment and multi-tasks of adaptive power-aware allocation scheme and propose the optimal task allocation algorithm under single task and the optimal voltage/frequency adjustment scheme under multi-tasks. Although the energy saving method under multi-tasks is studied, more attention is paid to voltage/frequency adjustment. For dynamic random access memory (DRAM)-based main memory subsystem is a major contributor to the energy consumption of mobile devices, Zhong et al. [27] propose direct read (DR). Swap by using NVMs byte addressability which guarantees zero memory copy for read-only requests when accessing a page in swap area. The research of [28] shows that the use of shared memory architecture in mobile devices can improve the cooperation among processors, accelerate the calculation of PCA (principal components analysis), and effectively reduce the energy of mobile devices. Khalid et al. [29] have proposed an OSCHED scheduling method in the case of unbalanced computing power of processors, which comprehensively considers the computing power of devices and the computing requirements of tasks to achieve load balancing of tasks among various processors. Hamano et al. [30] have proposed an energy saving method for dynamic scheduling. The task with the smallest energy delay product (EDP) is selected, and then, it is assigned to the corresponding processor, but the method considers that the power of the scheduled task is constant. Huang [31] points out that processing elements are idle when the required data are not received which will lead to the issue of low utilization of processing elements. Choi et al. [34] have proposed an estimated-execution-time (EET) scheduling to predict the remaining execution time of programs according to the remaining execution time of tasks and pointed out the deficiency of the alternate assignment (AA) scheduling, first free (FF) scheduling, and performance history (PH) scheduling in [32, 33]. That is, PH scheduling does not consider the remaining time of the application currently executed by each device, which will lead to overutilization of a single device. According to the methods proposed in [32–34], the scheduling tasks are extended to multiple tasks in [35, 36], and a 0-1 programming method is proposed to allocate tasks to solve the problem of excessive utilization of single processor. However, the results obtained by this method are greatly affected by parameter values.

In summary, although the energy saving research of heterogeneous systems has made great progress, there are still some deficiencies. In view of the existing problems and research deficiencies, this paper proposes HGES method to alleviate the problem.

## 3. Heuristics from 0-1 Programming

In [36], authors use 0-1 programming by formalizing the problem into formulas (1)–(6) to solve the low power scheduling problem in heterogeneous system. They assume that the currently available processor resources in the system are GPU_*i*_ (0 ≤ *i* ≤ *n*), CPU, and motherboard, and then the energy consumption of the system *E*_*system*_ can be expressed as the sum of the energy consumption of all GPUs (*E*_*GPU*_), CPU (*E*_*CPU*_), and motherboard (*E*_*Motherboard*_) in the system and further expressed as the product of their respective power (*P*_*GPU*_, *P*_*CPU*_, *E*_*Motherboard*_) and time (*T*). For a group of tasks to be scheduled on the same number of GPUs, the tasks to be scheduled will generate different sequences according to different scheduling algorithms without changing the task structure, but the power of a single task will not be changed; that is, the average power consumption of the task sequence to be scheduled remains unchanged. Therefore, the *E*_*system*_ can be further expressed as the product of average power consumption $\bar{P}$ and time *T* which can be expressed by

(1) $$\begin{array}{c} E_{System}=\sum_{i=1}^{n}E_{GPU_{i}}+E_{CPU}+E_{Motherboard}\\ =\left(\sum_{i=1}^{n}P_{{}_{GPU_{i}}}+P_{CPU}+P_{Motherboard}\right)\times T\\ =\left(\bar{P}+P_{CPU}+P_{Motherboard}\right)\times T. \end{array}$$

In order to minimize the energy of system when executing the program sequence, the average power consumption $\bar{P}$ and time *T* must be as small as possible. For different scheduling methods, the average power consumption is certain. Therefore, in order to minimize the energy consumption of the system, it is necessary to minimize the execution time *T*. When using 0-1 programming to solve this problem, we define the following symbols. Let *m* represent the number of GPU in systems; let *n* represent the number of programs to be processed in the system. Let *T*_*ij*_ represent the consumed time by the *j*th program running on the *i*th GPU (0 ≤ *j* ≤ *N*; 0 ≤ *i* ≤ *M*). Let *x*_*ij*_ represent assigning *i*th processor to complete the *j*th program, so the value of *x*_*ij*_ is as follows:

(2) $$\begin{array}{c} x_{ij}=\left\{\begin{array}{cc} 1, & \text{assign }ith\;GPU\text{ to execute }jth\text{ program}\\ 0, & \text{not assign }ith\;GPU\text{ to execute }jth\text{ program}. \end{array}\right.. \end{array}$$

The goal of the problem we solve is to choose a suitable combination that minimizes the time interval among each processor when executing tasks. We use the first processor as the baseline, so the objective function is the minimum executing time difference between other processors and the first processor. Therefore, the objective function to minimize the task execution time among processors can be shown in

(3) $$\begin{array}{c} f=m\sum_{j=1}^{n}T_{1j}x_{1j}-\sum_{k=2}^{m}\sum_{t=1}^{n}T_{kt}x_{kt}. \end{array}$$

According to the requirements of the problem, each program has only one processor to run, so we get the processor constraint as shown in (4).

(4) $$\begin{array}{c} \sum_{i=1}^{m}x_{ij}=1,\;j=1,2,\ldots ,n, \end{array}$$

(5) $$\begin{array}{c} Q\frac{\sum_{t=1}^{n}T_{1t}}{m}<=\sum_{j=1}^{n}T_{ij}*x_{ij},\;i=1,2,\ldots ,n. \end{array}$$

When assigning a task to a processor, the time to complete all tasks should be as equal as possible. We cannot unlimitedly reduce performance for saving energy, so we add constraint of performance to the objective function. Due to the randomness of the execution time of the program, it is not suitable for most scenes for allocating tasks to the each GPU in an equal time manner, respectively. In order to better adapt to the real environment, we allow unequal distribution of time on each GPU. For this, the total time of tasks allocated to a single processor in the system is not more than the average time that is calculated by total time of tasks divided by number of processors, so we use the performance tuning parameter *Q* to fulfill this purpose. The range of *Q* is 0.01–1. Considering above factors, we obtain the time constraint as shown in (5).

(6) $$\begin{array}{c} \left\{\begin{array}{c} \text{min}\;f=\;m\sum_{j=1}^{n}T_{1j}x_{1j}-\sum_{k=2}^{m}\sum_{t=1}^{n}T_{kt}x_{kt}\\ \begin{array}{c} s.t.\;\sum_{i=1}^{m}x_{ij} \end{array}\;=\;1\left(j=1,2,\ldots ,n\right)\\ Q\frac{\sum_{t=1}^{n}T_{1t}}{m}\;<=\;\sum_{j=1}^{n}T_{ij}*x_{ij}\left(i=1,2,\ldots ,n\right)\\ x_{ij}\;=\;0\text{ or }1 \end{array}\right.. \end{array}$$

In summary, when using 0-1 programming to solve above problem, it can be described as (6). In order to better understand it, let *m* be 4, *n* is 11, *T*_*ij*_ is consumed time by the 11 programs running on the 4 GPUs, and *x*_*ij*_ assigns *i*th processor to complete the *j*th program. The constraint *x*_*ij*_ = 0 or 1 and ∑_*i*=1_^*m*^*x*_*ij*_=1(*j*=1,2,…, *n*) guarantee each of 11 tasks assigned to only one GPU; the constraint *Q*∑_*t*=1_^*n*^*T*_1*t*_/*m* < =∑_*j*=1_^*n*^*T*_*ij*_*∗x*_*ij*_(*i*=1,2,…, *n*) guarantees feasible solutions under different parameters *Q*. The objective function ensures that the optimal solution can be found in the feasible solution.

Figure 1 shows the impact of the *Q* parameter changes on the result of 0-1 programming when 20 tasks are scheduled. The abscissa is the value of *Q* parameter, and the ordinate represents energy consumption. It can be seen from the figure that with gradual increase in the value of *Q*, the energy consumption is gradually reduced. Therefore, the reasonable value of *Q* has a great influence on the energy consumption of the system. Since the solution obtained by 0-1 programming is greatly affected by the *Q* parameters, unreasonable *Q* parameter often results in nonhigh-quality solution for solving the problem. In the process of solving 0-1 programming, the feasible solution satisfying the constraint conditions is first calculated, and then the optimal solution satisfying the objective function is considered. Analyzing the solution obtained, we find that there are time-consuming tasks assigned to each processor, regardless of the value of the *Q* parameter.  Figure 2 shows the result of assigning tasks using 0-1 programming with a *Q* parameter of 0.4 (sub-figure (a)) and a *Q* parameter of 0.9 (sub-figure (b)). It can be seen from the figure that different *Q* parameters affect the scheduling results. The reason for this phenomenon is that the obtained feasible solution must meet the constraint conditions, and the time-consuming tasks will be evenly allocated to each processor so that the obtained feasible solution minimizes the objective function.

Based on the inspiration of the 0-1 programming, we should first seek the tasks satisfying the constraint conditions and then select the tasks within them which can minimize the objective function. In the process of finding tasks that satisfy the constraints, the execution time of task allocated to each processor should be made as equal as possible to minimize the objective function. Therefore, the cumulative task's execution time of processors should be considered when assigning tasks. For the tasks with long execution time have a greater impact on the constraint conditions, so the tasks with longer execution time should be allocated first. In allocating tasks to suitable processors that satisfy the objective function, the greedy method is used to comprehensively consider the total time of the processor's allocated tasks and the time and energy of the tasks to be allocated to find processors that meet the objective function. After the tasks with longer execution time are assigned, the tasks with smaller execution time are allocated according to the same rules.

## 4. HGES Approach

Inspired by the above 0-1 programming, we call the method to solve this problem as heuristic and greedy energy saving approach (HGES). The main idea first assigns all tasks to each processor; secondly, tasks are divided into two parts according to the execution time in each processor. The tasks with long execution time in each processor are assigned first. When a task is assigned, then it will be deleted from all task list of other processors to be allocated. This process is repeated until all tasks with long execution time are allocated; thirdly, the task with short execution time is assigned to each processor, and when the task is assigned, it will be deleted from all task list of other processors to be allocated. This process is repeated until the short execution tasks are assigned. The allocation rule is to select the task with the smallest product of the processor's cumulative time and the energy consumption of the corresponding task to be allocated among the *K* smallest cumulative execution time of *m* processors.

For scheduling, the scheduling parameters of *P* tasks should be obtained first; therefore, we establish a two-dimensional array GPU_Time_Energy_*i*[*P*] for each processor *i* to store the time and energy consumption of tasks, which are, respectively, GPU_Time_Energy_*i*[*P*][0] and GPU_Time_Energy_*i*[*P*] [1]. The variable *AccumPer*_*i* is used to store the sum of the execution time of the assigned tasks to each processor *i*. *AVE*_*i*_ and *SD*_*i*_ are used to estimate the average execution time and the corresponding standard deviation of each processor *i* under *n* tasks, and equation (7) is used to calculate the criterion *Crit*_*i*_ to distinguish the length of execution time. *Crit*_*i*_ is used to separate tasks that affect performance constraints. The tasks with a long execution time corresponding to the processor number *i* are put in the *Th*_*i* array, and the remaining tasks are put in the *Tm*_*i* array. Each *Th*_*i* array is sorted in descending order, and they are scheduled according to greedy method. The steps of greedy method are as follows. Firstly, select the *K* processors with the smallest cumulative sum of time, and secondly, assign the task to the processor with the smallest product of the cumulative time of *K* processor and the energy consumption of the corresponding task to be allocated. After the corresponding *Th_i* of each processor is scheduled, the same rules are used to schedule *Tm*_*i*.

(7) $$\begin{array}{c} {\text{Crit}}_{i}=AVE_{i}+SD_{i}. \end{array}$$

According to the above ideas, Figure 3 shows the flow of the HGES method. The specific steps are as follows:

  Step 1: All *P* tasks are allocated to each processor *i*, and the corresponding time and energy are, respectively, stored in GPU_Time_Energy_*i*[*P*][0] and GPU_Time_Energy_*i*[*P*] [1]; the performance accumulator *AccumPer*_*i* is initialized to 1 for each processor *i* and the task allocation sequence *AllocTask*_*i* to null.
  Step 2: Average execution time AVEi and the standard deviation SDi of the P tasks in each processor *i* are calculated.
  Step 3: Execution time of tasks that are higher than the *Crit*_*i*_ in the GPU_Time_Energy_*i*[*P*][0] of each processor *i* is stored in *Th*_*i*, and they are sorted in descending order. The sorted task index list is *Sort*_*Th*_*i*[*pth*_*i*]. The list of remaining tasks is *Tm*_*i*[ *ptm_i*]; *pth_i* and *ptm_i* are the subscripts of the corresponding task list.
  Step 4: Determine whether the assignment of *P* tasks is complete. If complete, terminate the algorithm; if not, the *Sort_Th_i* or *Tm_i* corresponding to the *K* processors with the minimum cumulative task execution time is selected. Calculate *K* values according to the following steps. Determine whether *Sort_Th_i* has been allocated completely, that is, whether *pth*_*i* is greater than the maximum subscript of *Sort_Th_i*, *Maxpth*. If it is less, judge whether the current task has been allocated, that is, whether *GPU_Time_Energy_i*[*Sort_Th_i*[*pth_i*]][0] is equal to 0. If it is equal to 0, that means that the task has been allocated to other processors, and *pth_i* needs to be increased by one to determine whether the next task is allocated; if it is not equal to 0, calculate the product of the accumulated time of processor and the corresponding power consumption of current task, namely, *AccumPer_i∗GPU_Time_Energy_i*[*Sort_Th_i*[*pth_i*]] [1], and assign the calculation result to *TTE_i*. If *pth_i* is greater than the maximum subscript *Maxpth* of *Sort_Th_i*, it means that *Sort_Th_i* has been allocated completely and it is necessary to determine whether *Tm_i* has been allocated completely, that is, whether *ptm_i* is greater than the maximum subscript of *Tm_i*, *Maxptm*. If it is greater, it indicates *Tm_i* has been allocated completely and all tasks in the processor have been allocated. Assign the *Max_Value* value to *TTE_j* so that it does not participate in task allocation. If it is less than, judge whether the task has been allocated, that is, whether *GPU_Time_Energy_j*[*Tm_j*[*ptm_j*]][0] is equal to 0. If it is equal to 0, it means that the task has been allocated to other processors, and *ptm_i* needs to be increased by one to determine whether the next task is allocated. If it is not equal to 0, calculate the product of the accumulated time of processor and the corresponding power consumption of current task, namely, *AccumPer_i∗GPU_Time_Energy_i*[*Tm_j*[*ptm_j*]][0], and assign the calculation result to *TTE_j*.
  Step 5: Among *K TTE_i* or *TTE_j*, select the processor number *minENumGPU* corresponding to the smallest value, and determine whether *minENumGPU* comes from *Th_i*. If so, accumulate corresponding time to the corresponding processor; that is, add *GPU_Time_Energy_minENumGPU*[*Th_i*[*pth_i*]][0] to *AccumPer_minENumGPU*. Assign the corresponding task to the list of the corresponding processor, namely, *TaskAlloc_minENumGPU* = *Th_i*[*pth_i*]. This task will not be considered in the next allocation, and the execution time of all processors corresponding to this allocated task will be assigned to zero; that is, set *GPU_Time_Energy_minENumGPU* [*Th_i*[*pth_i*]][0] to 0. Then, add one to the corresponding subscript to prepare for the next task; that is, add one to *pth_i*. At this point, one task has been assigned. Therefore, the parameter Counter indicating the number of assigned tasks is added by one; if *minENumGPU* comes from *Tm_i*, the processing process is the same as that of the task from *Th_i*. The difference is that the processed data come from *Tm_i*.

The pseudocode of the specific HGES method is shown in Algorithm 1. The input of Algorithm 1 is *P* tasks and *NumGPU* processors; the output is program sequence to be executed on each GPU, *AllocTask_NumGPU*. In the first line of Algorithm 1, the execution time, power consumption, average execution time, and standard deviation of execution time of *P* tasks on each GPU are obtained. Lines 2 to 10 use average execution time and standard deviation to filter tasks with long execution time and tasks with short execution time; tasks with long execution time for each processor are placed in *Th_i*, and tasks with short execution time are placed in *Tm_i*. Line 11 gets the total number of long execution time and short execution time of tasks. The 12th to 14th lines sort *Th_i*, and the sorted *Th_i* is represented by *Sort_Th_i*. Lines 15 through 27 assign *P* tasks according to the allocation rules. Among them, the 16th line adopts the bubble sorting idea to select *K* processor with the smallest cumulative time. Algorithm 2 is its specific implementation, which can be completed by once traversing. The return value is *K_GPUIndex* for the corresponding *K* processor number. The 17th line gets GPU number, task index, and the task index in array *Th* or *Tm* array corresponding to the smallest product of the *K* accumulated time of GPU, and the energy of current task in *Sort_Th_i* or *Tm_i*. Algorithm 3 is its specific implementation. The return value *ret_GPUIndex* is the processor to be allocated, *ret_taskindex* is the subscript number of the task in *Sort_Th_i* or *Tm_i*, and *thortm* indicates whether *ret_taskindex* is in *Sort_Th_i* or *Tm_i*. Lines 18 to 21 represent that *ret_taskindex* is in *Sort_Th_i* and the task is assigned to the corresponding processor (line 19). Line 20 accumulates the assigned task execution time to the execution time accumulator of the corresponding processor. Line 21 clears the time of the assigned task corresponding to all processor lists, indicating that the task has been assigned to the corresponding processor and cannot be assigned to other processors in the next assignment. Lines 22–26 are the *ret_taskindex* in *Tm_i*, and the processing is similar to lines 18–21. The difference is that the task to be processed is in *Tm_i*. The 28th line returns the obtained result.

Algorithm 2 uses the bubble sorting idea to select the *K* processor number with the smallest cumulative execution time. The input is the cumulative execution time of each processor; the output is the *K* processor number with the smallest cumulative execution time. Line 1 initializes related variables. Lines 2–8 traverse the cumulative time of each processor; lines 3–7 are used to get *K* return values; lines 4–6 filter the *NumGPU* − *K* processor number of the maximum value, where the maximum value is stored in the *high* variable; line 9 returns the remaining *K* processor number.

Algorithm 3 gets the task number and processor number with the smallest product of accumulated time and energy of its task among the *K* processor output by Algorithm 2. Lines 1–12 process the tasks in *Sort_Th_i* corresponding to *K* processors. Lines 2–7 select the subscript of the unassigned task in *Sort_Th_i*. Lines 8–11 calculate the product of the cumulative time of the corresponding processor and the energy of the task corresponding to the subscript obtained from lines 2–7. Lines 13–23 deal with the tasks in *Tm_i*. Lines 14–19 select the subscript of the unassigned task in *Tm_i*. Lines 20–22 calculate the product of the energy consumption of the task which is pointed by the subscript obtained by lines 14–19 and the cumulative time of the corresponding GPU. The 24th line calculates the product of the energy consumption of current task and the cumulative time in the *K* *−* 1 GPU. Lines 25–30 select the processor number with the smallest product among the *K* processors. Lines 31–36 return the processor number, task index, and whether the task is in *Sort_Th_i* or *Tm_i*.

For the efficiency of HGES, in the case of problem size *n*, the time complexity of acquiring task time, power consumption, *AVE*_*i*_, and *SD*_*i*_ is *O*(*n*); the time complexity of filtering feasible solutions is *O*(*NumGPU∗n*); the time complexity of sorting *Th_i* is *O*(*n*log*n*); the time complexity of assigning tasks according to heuristic and greedy methods is *O*(2*∗NumGPU∗n*). Generally, the number of processors in the system *NumGPU* is often constant. In summary, the time complexity of the HGES method is *O*(*n*log*n*).

## 5. Experiment

In order to verify the effectiveness and adaptability of HGES method, we choose two platforms for verification, named platform A and platform B. The hardware experimental environment of platform A includes i5-7500 CPU and 3 NVIDIA GeForce GTX 1060 graphics cards. The system memory is 8 GB. The architecture of GTX 1060 card is Pascal. GTX 1060 has 6 GB GPU memory and 10 SMs (streaming multiprocessors), each containing 128 CUDA (Compute Unified Device Architecture) cores, 1280 CUDA cores in total. Single card can provide 4.4 TFLOPS (floating point operations per second) computing capabilities. The hardware experimental environment of platform B includes i5-7500 CPU and 3 NVIDIA GeForce GTX 2080 graphics cards. The system memory is 8 GB. The architecture of GTX 2080 card is Turing. GTX 2080 has 8 GB GPU memory and 46 SMs, each containing 64 CUDA cores, 2944 CUDA cores in total. Single card can provide 10.6 TFLOPS computing capabilities. The software experimental environment is Windows 10, VS2015 and CUDA9.2. All the hardware and software experimental environments are listed in Table 1.

For better verified HGES, six typical CUDA benchmark tasks are selected to better verify the algorithm and different input sizes and different numbers are selected to simulate. These benchmarks are, namely, matrix multiplication (MM), histogram (HG), scalar products (SP), BlackScholes (BS), vectorAdd (VA), and mergeSort (MS). Their specific parameters are shown in Table 2.

For getting the energy, HIOKI 3334 AC/DC power meter is selected to measure the energy of the system. For the number of tasks is less than that of GPUs, PH and EET methods almost all degenerate into FIFO methods, resulting in a little performance difference. For this purpose, these experiments are unnecessary to be done. The HGES approach in this paper is implemented as follows. Firstly, the pseudocode in Algorithm 1 through 3 is running in VS2015. Secondly, we reprogram the task order based on the output result of HGES by the first step. For measuring the energy, the energy consumptions of the algorithm itself and the energy consumption of the running task are two parts of the approached energy, so we, respectively, record them as Energy 1 and Energy 2; finally, Energy 1 adds Energy 2 are the energy of HGES.

Figures 4 and 5 show the time difference between HGES and 0-1 programming in scheduling results of platforms A and B under different parameters and different numbers of tasks. The abscissa in the figures represents the values of different *Q* parameters under 0-1 programming, and the ordinate represents time. The subfigures (a), (b), (c), and (d) show the time difference of 10, 20, 40, and 80 tasks, respectively. The red star in each figure represents the time difference of the scheduling results obtained by the HGES method. From the overall perspective of Figures 4 and 5, as the *Q* parameter gradually approaches 1, the time difference of the scheduling results gradually decreases; when the parameter *Q* is set to 0.9, the time difference of the scheduling results is the smallest; when the *Q* parameter is 1, (a), (b), (c), and (d) in Figures 4 and 5 cannot get the optimal solution. The trend in these figures shows that the optimal solution obtained by the 0-1 programming is affected by the *Q* parameter. The smaller the *Q* value, the worse the scheduling effect. When the *Q* is 1, there is no solution. Compared with 0-1 programming, the time difference of HGES under different tasks in different platforms is the smallest. In Figures 4 and 5, when the number of scheduling tasks is 10 and the *Q* sets 0.1, the time difference of 0-1 programming is 5.22 s in Figure 4 and 2.259 s in Figure 5. When *Q* sets 0.9, the time difference is 0.573 s in Figure 4 and 0.3667 s in Figure 5. The time difference of HGES is 0.445 s in Figure 4 and 0.3424 s in Figure 5 under the 10 scheduling tasks. When the scheduling quantity is 20 tasks, the time difference of 0-1 programming is 7.86 s in Figure 4 and 5.417 s in Figure 5 when *Q* is 0.1. When *Q* is 0.9, the time difference is 0.536 s in Figure 4 and 0.361 s in Figure 5. The time difference of HGES is 0.365 s in Figure 4 and 0.233 s in Figure 5. In the case of scheduling 40 tasks, the time difference of 0-1 programming is 9.709 s in Figure 4 and 7.367 s in Figure 5 when *Q* is 0.1. When *Q* is 0.9, the time difference is 0.974 s in Figure 4 and 0.756 s in Figure 5. The time difference of HGES is 0.271 s in Figure 4 and 0.173 s in Figure 5. When scheduling 80 tasks, the time difference of 0-1 programming is 22.8 s in Figure 4 and 12.3 s in Figure 5 when *Q* is 0.1. When *Q* is 0.9, the time difference is 2.53 s in Figure 4 and 2.1 s in Figure 5. The time difference of HGES is 0.203 s in Figure 4 and 0.129 s in Figure 5. In Figures 4 and 5, the results of HGES method are similar under different numbers of scheduling tasks. From the experimental data, HGES has obvious effect on reducing the time difference when scheduling tasks.

Figures 6 and 7 show the energy consumption comparison between HGES and 0-1 programming in scheduling results of platforms A and B under different parameters and different numbers of tasks. The abscissa in figures represents the different values of *Q* parameters under the 0-1 programming, and the ordinate represents the energy consumption. Sub-graphs (a), (b), (c), and (d) show the energy consumption of HGES and 0-1 programming under 10, 20, 40, and 80 tasks, respectively. Each red star in the sub-graph represents the energy of the scheduling results obtained by HGES method. From the overall perspective of Figures 6 and 7, as the *Q* parameter gradually approaches 1, the energy is gradually reduced; when the parameter *Q* sets to 0.9, the energy consumption is the smallest. When the *Q* parameter is 1, the 0-1 programming in sub-graphs (a), (b), (c), and (d) cannot be solved. The trend in the figure shows that the optimal solution obtained by the 0-1 programming is affected by the *Q* parameter. The larger the *Q* value, the lower the energy consumption. When the *Q* is 1, there is no solution. Compared with 0-1 programming, HGES method consumes the least energy consumption under different tasks in Figures 6 and 7. In the experiment, when the number of scheduling tasks is 10 and *Q* is 0.1, the energy of 0-1 programming is 456.21 J in Figure 6 and 323.6 J in Figure 7. When *Q* is 0.9, the energy is 321.13 J in Figure 6 and 237.5 J in Figure 7. The energy of HGES is 313.12 J in Figure 6 and 235.4 J in Figure 7. When 0-1 programming schedules 20 tasks and the *Q* is 0.1, its energy is 596.16 J in Figure 6 and 427.2 J in Figure 7. When *Q* is 0.9, its energy is 418.74 J in Figure 6 and 318.5 J in Figure 7. The energy of HGES under 20 tasks is 393.73 J in Figure 6 and 291.7 J in Figure 7. When 0-1 programming schedules 40 tasks and *Q* is 0.1, its energy is 1,453.42 J in Figure 6 and 1,044.4 J in Figure 7. When *Q* is 0.9, its energy is 1,012.82 J in Figure 6 and 761.9 J in Figure 7. The energy consumption of HGES under 40 tasks is 945.84 J in Figure 6 and 703.3 J in Figure 7. When 0-1 programming schedules 80 tasks and *Q* is 0.1, its energy is 1,801.86 J in Figure 6 and 1278.5 J in Figure 7. When *Q* is 0.9, its energy is 1,227.45 J in Figure 6 and 909.9 J in Figure 7. The energy consumption of HGES under 80 tasks is 1,140.76 J in Figure 6 and 848.6 J in Figure 7. From the experimental data, HGES is more effective than 0-1 programming in energy saving.

Figures 8 and 9 show the performance comparison between HGES and the 0-1 programming itself. The abscissa in the figure represents the different *Q* parameters of 0-1 programming, and the ordinate represents the time. Subgraphs (a), (b), (c), and (d) show the time of HGES and 0-1 programming under 10, 20, 40, and 80 tasks, respectively. Each red star in the sub-graph represents the time of the HGES. Looking at each figure as a whole, as the *Q* value increases, the time consumed by 0-1 programming increases. In the sub-figure (b) and (d) of Figures 8 and 9, as the *Q* value increases, the time-consuming effect of 0-1 programming is the most significant. This phenomenon also appears in the sub-figure (c) of Figure 9. In the sub-figure (a) of Figures 8 and 9, the time consumed by 0-1 programming is relatively flat. In the subfigure (c) of Figure 8 when *Q* values are 0.1 to 0.4 and 0.6–0.8, the consumed time tends to increase. When *Q* values are 0.4 to 0.6 and 0.9, the time consumption decreases. However, the consumed time of 0.9 is more than that of 0.4 to 0.6. The HGES is the least time-consuming in all experiments. In the case of 10 tasks in Figure 8, the minimum consumed time of 0-1 programming is 0.011 s when *Q* is 0.2; the maximum consumed time is 0.031 s when *Q* is 0.1. The consumed time of HGES is 0.001 s, which improves the processing speed, respectively, 11 times and 31 times compared with that of 0-1 programming when *Q* is 0.2 and 0.1. In Figure 9, the consumed time of HGES is 0.001 s, which improves the processing speed, respectively, 10 times and 23 times compared with that of 0-1 programming when *Q* is 0.2 and 0.9. In the case of 20 tasks in Figure 8, the minimum consumed time of 0-1 programming is 0.03 s when *Q* is 0.1. The maximum consumed time is 0.9146 s when *Q* is 0.9. The consumed time of HGES is 0.0016 s, which improves the processing speed, respectively, 18.75 times and 517.62 times compared with that of 0-1 programming when *Q* is 0.1 and 0.9. In Figure 9, the consumed time of HGES is also 0.0016 s, which improves the processing speed, respectively, 37 times and 585 times compared with that of 0-1 programming when *Q* is 0.1 and 0.7. In the case of 40 tasks in Figure 8, the minimum consumed time of 0-1 programming is 0.103 s when *Q* is 0.1. The maximum consumed time is 0.346 s when *Q* is 0.9. The consumed time of HGES is 0.019 s, which improves the processing speed, respectively, 5.42 times and 18.21 times compared with that of 0-1 programming when *Q* is 0.1 and 0.9. In Figure 9, the consumed time of HGES is also 0.019 s, which improves the processing speed, respectively, 5.6 times and 50.5 times compared with that of 0-1 programming when *Q* is 0.4 and 0.9. In the case of 80 tasks in Figure 8, the minimum consumed time of 0-1 programming is 0.402 s when *Q* is 0.1. The maximum consumed time is 2.368 s when *Q* is 0.7. The consumed time of HGES is 0.047 s, which improves the processing speed, respectively, 8.55 times and 50.38 times compared with that of 0-1 programming when *Q* is 0.1 and 0.7. In Figure 9, the consumed time of HGES is 0.046 s, which improves the processing speed, respectively, 11.1 times and 21.2 times compared with that of 0-1 programming when *Q* is 0.1 and 0.4. It can be seen from the experimental data that HGES has a great advantage in processing speed. Figures 10 and 11 show the energy comparison between HGES and the 0-1 programming. The trend shown in Figures 10 and 11 is similar to that in Figures 8 and 9, and it will not be repeated here.

Figures 12 and 13 show the comparison of allocation time of HGES and 0-1 programming with different parameters in each processor. The abscissa in figures represents the various methods, which are the different parameters of 0-1 programming and the HGES method; the ordinate is the ratio of processor allocation time. It can be seen from figures that with the increase in the value of *Q* parameter, the more balanced the execution time of each processor is, and there is no solution when *Q* is taken as 1. When *Q* is 0.9 in Figure 12, the proportion of task execution time of each processor is 30%, 33.07%, and 37.59%, respectively. The HGES method makes the proportion of task execution time of each processor to be 33.69%, 33.08%, and 33.23%, respectively. When *Q* is 0.9 in Figure 13, the proportion of task execution time of each processor is 30%, 30.03%, and 39.97%, respectively. The HGES method makes the proportion of task execution time of each processor to be 33.69%, 33.08%, and 33.23%, respectively. In conclusion, HGES is more balanced in task allocation than that of 0-1 programming.

Figures 14 and 15 show the performance and energy comparison of PH, EET, and HGES under 80 tasks. The abscissa of (a) and (b) in each figure is the different scheduling methods. The ordinate in (a) represents time, and the ordinate in (b) represents energy consumption. Sub-figures (a) in Figures 14 and 15 show the time of each method; from figures, we can see HGES method is more balanced than PH and EET methods in assigning tasks. In Figure 14, the time difference of executing tasks between the processor with the highest time and the processor with the lowest time of PH is 9.52 s; the time difference of executing tasks between the processor with the highest time and the processor with the lowest time of EET is 5.39 s; the time difference of executing tasks between the processor with the highest time and the processor with the lowest time of HGES is 0.2036 s. In Figure 15, the time difference of executing tasks between the processor with the highest time and the processor with the lowest time of PH is 6.018 s; the time difference of executing tasks between the processor with the highest time and the processor with the lowest time of EET is 3.518 s; the time difference of executing tasks between the processor with the highest time and the processor with the lowest time of HGES is 0.13 s. These show that the HGES is more effective than PH and EET in assigning tasks. Sub-figures (b) in Figures 14 and 15 show the energy of each method and its executing tasks. From figures, we can see HGES consumes the least energy in scheduling tasks than that of other methods. In Figure 14, PH consumes 1465.20 J energy; EET consumes 1355.61 J energy; HGES consumes 1140.76 J energy. The HGES saves 22.14% energy than that of PH and 15.84% energy than that of EET. In Figure 15, PH consumes 1057.16 J energy; EET consumes 986.82 J energy; HGES consumes 848.65 J energy. The HGES saves 19.72% energy than that of PH and 14.01% energy than that of EET. In conclusion, HGES is more effective than PH method and EET in task allocation and energy saving.

## 6. Conclusion

Today's society is increasingly advocating sustainable development, and the energy consumption of heterogeneous systems has become an important issue that people are concerned about. This paper studies the energy saving problems of heterogeneous systems composed of multiple identical GPUs, analyzes the reasons for their energy consumption, summarizes the characteristics of the solution obtained by the 0-1 programming, lists the shortcomings of the current method, and adopts heuristic and greedy methods to solve the energy saving problem of heterogeneous systems composed of multiple identical GPUs. Based on this, the HGES scheduling method is proposed. Firstly, HGES assigns all tasks to each processor in the system, and the average value and standard variance of execution time are calculated. Then, the tasks are divided into high-value part and low-value part according to the average and standard variance value. The high-value part is allocated first according to the accumulated time of each processor, and then the low-value part is allocated after the allocation of the high-value part. In order to verify the effectiveness and rationality of HGES, experiments were conducted with different numbers and different input tasks and different methods are used to compare. The experimental results show that the HGES has better effect on performance and energy saving.

## Figures and Tables

**Figure 1:** The influence of *Q* parameter on optimization results.

**Figure 2:** Patterns of 0-1 programming for assigning tasks.

**Figure 3:** Flowchart of HGES method.

**Figure 4:** Comparison of time difference between HGES and 0-1 programming in scheduling results of platform A.

**Figure 5:** Comparison of time difference between HGES and 0-1 programming in scheduling results of platform B.

**Figure 6:** Energy comparison between HGES and 0-1 programming in scheduling results of platform A.

**Figure 7:** Energy comparison between HGES and 0-1 programming in scheduling results of platform B.

**Figure 8:** Performance comparison of HGES and 0-1 programming itself of platform A.

**Figure 9:** Performance comparison of HGES and 0-1 programming itself of platform B.

**Figure 10:** Energy comparison between HGES and 0-1 programming itself in platform A.

**Figure 11:** Energy comparison between HGES and 0-1 programming itself in platform B.

**Figure 12:** Comparison of allocation time of HGES and 0-1 programming with different parameters of platform A.

**Figure 13:** Comparison of allocation time of HGES and 0-1 programming with different parameters of platform B.

**Figure 14:** Performance and energy comparison of HGES, PH, and EET in platform A.

**Figure 15:** Performance and energy comparison of HGES, PH, and EET in platform B.

**Algorithm 1:** The pseudocode of HGES.

**Algorithm 2:** Selecting *K* GPU number with the smallest cumulative execution time.

**Algorithm 3:** Getting the task and GPU number with the smallest product of accumulated time and energy of its task.

**Table 1:** The hardware and software environments.

	Hardware platform A		Hardware platform B	Software environment
CPU		I5-7500	I5-7500	Windows10 + VS2015 + CUDA 9.2
System memory		8 GB	8 GB	
GPU		GeForce GTX 1060	GeForce GTX 2080	
GPU memory		6 GB	8G	
GPU architecture		Pascal	Turing	
SM		10	46	
CUDA cores per SM		128	64	

**Table 2:** Benchmark tasks.

Application	Description	Input data range
Matrix multiplication (MM)	Using tiling approach to make use of shared memory to ensure data reuse	200^*∗*^5120 through 8100^*∗*^68400
Histogram (HG)	64-bin histogram calculation of arbitrary-sized 8-bit data array	64 M through 2048 M
Scalar products (SP)	Scalar products of a given set of input vector pairs	16 M through 384 M
BlackScholes (BS)	Evaluation fair call and put prices for a given set of European options by Black–Scholes formula	20000000 through 98000000
vectorAdd (VA)	Implements element by element vector addition	20 M through 400 M
mergeSort (MS)	Bottom-level merge sort (binary search-based)	2 M through 32 M

## Data Availability

The data used to support the findings of this study are available from the corresponding author upon request.
